# Analysis of the Association between Teachers' Classroom Teaching Behaviors and Students' Knowledge Acceptance Based on Psychological Data Analysis

This article has been retracted.

**DOI:** 10.1155/2022/2661398

**Published:** 2022-06-13

**Authors:** Tianjin Yao, Xiuye Yang

**Affiliations:** ^1^Faculty of Psychology and Education, Universiti Malaysia Sabah, Kota Kinabalu 88400, Malaysia; ^2^School of Economics and Management, Huanghe Jiaotong University, Jiaozuo Henan 454950, China; ^3^Department of Art and Design, Huanghe Jiaotong University, Jiaozuo Henan 454950, China

## Abstract

This paper adopts the method of psychological data analysis to conduct in-depth research and analysis on the correlation between teachers' classroom teaching behaviors and students' knowledge acceptance. Firstly, this paper proposes a health factor prediction model, which is specifically divided into clustering and then classification model and a clustering and classification synthesis model. The classroom learning process is coded, sampled, and quantified to obtain data on students' learning behaviors, and a visualization system based on classroom students' learning behaviors is designed and developed to record and analyze students' behaviors in the classroom learning process and grasp students' classroom learning. These two models use algorithms to fine-grained divide the dataset from the perspective of subject users and mental health factors, respectively, and then use decision tree algorithms to classify and predict the mental health factor information by the subject user base information. Second, based on the collected datasets, we designed comparison experiments to validate the clustering-then-classification model and the integrated clustering-classification model and selected the optimal model for comparison. Teachers should increase effective praise and encouragement behaviors; teachers should increase meaningful teacher-student interaction behaviors; teachers should be proficient in teaching media technology to reduce unnecessary time wastage. Strategies to enhance teachers' TPACK include enriching teachers' knowledge base of CK, TK, and PK; developing teachers' integration thinking; and enriching teachers' types of activities for integrating technology.

## 1. Introduction

In the context of education informatization, the integration of education and technology has promoted the great development of education. Smart education is the development direction of education today. To realize the development of wisdom in education, there are new requirements for the main places of classroom teaching. The smart classroom is precisely the form of the classroom created to promote the wisdom of education [1]. With the development of smart education, the smart classroom is constantly optimized and plays an important role in improving the quality of classroom teaching and optimizing the teaching effect. With the current change of educational philosophy, there are many problems in the traditional classroom in the process of promoting the development of educational wisdom [2]. Through in-depth analysis of the differences between different individuals, we can understand the psychology and behavior of individuals and help scientists understand the laws of group psychology and behavior. As one of the three main subjects of education in China, the importance of learning English is self-evident. Middle school English is at the stage of bridging elementary English and high school English and therefore plays an important role in the learning of English. Whether it is the smart classroom or the traditional classroom, there are still certain problems and needs in the classroom teaching of school English [3]. This study will specify the background of the research from the following three aspects. Teachers pay attention to the explanation of book knowledge and cannot combine what they learn with real life, so students' understanding of knowledge is abstract. Students cannot flexibly apply what they have learned, and their understanding of knowledge is not deep enough [4]. The traditional classroom teaching method and teaching means are relatively single, and the teacher occupies a dominant position in the classroom, which inhibits students' learning autonomy and learning initiative. In the teaching process, the teacher's simple explanation seems more boring and cannot stimulate students' interest in learning, and students lack the initiative of learning [5]. The use of teaching media and media function is single, using multimedia mainly to display courseware and play audio and video the classroom is still teacher lecture-oriented; teaching media only play a small role. In addition, in traditional classroom teaching, teachers set teaching objectives, design teaching contents, and arrange teaching schedules based on the overall level of the class [6–10]. Therefore, the support of relevant research is needed to help teachers summarize the characteristics. Teachers can analyze and evaluate their own teaching behavior and teacher TPACK by referring to relevant research conclusions and reflect on the current problems. Teachers do not consider the learning differences among students and their learning demands, ignoring the existence of individual students' differences and failing to promote students' personalized development.

Smart education meets students' personalized development, the teaching process of smart education changes from static to dynamic, and smart education focuses on students' overall development. These characteristics of wisdom education make teachers must have a more solid foundation and more professional skills, which is a deeper requirement for teachers' professionalism. Teachers' teaching behavior is the outward expression of teachers' knowledge, teachers' quality, and teachers' ability and the outward manifestation of teachers' professionalism [11]. To follow the development trend of the times and promote the teaching effectiveness of English in the smart classroom, teachers should make changes. Teachers should change their attitude toward the integration of technology and subjects and actively explore suitable methods of integrating technology and subjects in the classroom according to the actual teaching situation. In addition, teachers need to have a general understanding of their teaching behaviors and TPACK in the smart classroom, and they need to identify the gap between their current level and the required level [12–18]. Therefore, teachers need the support of relevant studies to help them summarize the characteristics, and they can analyze and evaluate their teaching behaviors and teacher TPACK by drawing on the findings of relevant studies to reflect on the current problems. According to the strategies of the study, they can choose appropriate opinions and suggestions to solve their teaching problems in a targeted way and improve the quality of teaching for professional development [19].

However, making full use of some comprehensive key indicators of the psychological assessment system can not only grasp the psychological development trend of the test subjects but also provide some effective decision-making assistance for mental health counseling work [20]. Teachers' teaching behavior is the external manifestation of teachers' knowledge, quality and ability, and the external manifestation of teachers' professional quality. A subject can be assessed daily, monthly, or annually through the psychological assessment system, and the data of the assessment results are so numerous that managers cannot grasp the mental health data of the subject group in detail, and data mining technology brings solutions to the complicated data problems. Using network data, we can break through the limitations of traditional psychological research and through more representative data collection samples and in-depth analysis of the differences between different individuals, to understand the psychology and behavior of individuals and help scientists understand the laws of group psychology and behavior. It helps teachers adjust their teaching methods and strategies as well as gain practical knowledge through reflection, which helps to promote the quality of classroom teaching. It provides reference and reference for the rational arrangement of information-based classroom teaching activities.

## 2. Method

### 2.1. Design

Constructivist theory is based on a student-led and teacher-led form of teaching, in which the task of students is to construct meaning, while the teacher's task is no longer simply to impart knowledge, but to inspire students to construct meaning in the right direction [21]. In a student-led and teacher-led teaching format, teachers should take the cultivation of students' interest in learning as the base and motivate students to actively engage in meaning construction to fundamentally promote students' learning. Therefore, teachers need to not only standardize classroom teaching behaviors.

The proposed interaction analysis system is widely used in the study of teacher-student verbal interaction and has a high degree of universality, but because the system was proposed earlier, it cannot be fully matched with the current study, so researchers should modify it scientifically according to the actual situation [22]. Among them, the rules for coding classroom behaviors mentioned in the Flanders interaction analysis system are to code the samples in 1 unit of 3 seconds, but teaching behaviors cannot last for 3 seconds in the real teaching process, which may result in redundant continuous units and is not conducive to the smooth conduct of the study. Therefore, this study slightly modified Flanders' interaction analysis system when developing the classroom teaching behavior coding form and used a complete teaching behavior as a duration unit to ensure its completeness. In addition, teachers' classroom teaching behaviors are closely related to students' classroom behaviors; therefore, this study added the dimension of students to the coding of classroom teaching behavior classification, as shown in Table 1.

First, effective teaching is an ideal vision of teaching that is formed by people under the domination of specific teaching values [23]. The process of English teachers pursuing the effectiveness of teachers' teaching behaviors in the context of blended teaching is also the process of pursuing how to promote students' learning and how to promote learning, which coincides with the concerns of effective teaching theory. It is impossible to study the effectiveness of English teachers' teaching behaviors in the context of blended teaching in isolation from the concept of effective teaching. Secondly, in the age of information technology, the cultivation of higher-order thinking skills is also particularly important, and teachers can promote the cultivation of students' higher-order thinking skills through the effectiveness of online and offline teaching behaviors in the context of blended teaching. This is also consistent with the view of teaching goals pursued by effective teaching theory. The use of teaching media and media functions is single. The use of multimedia is mainly to display courseware and play audio and video. In fact, the classroom is still mainly taught by teachers, and teaching media only play a small role.

In plain language, data mining is the mining of knowledge from data. The acquired knowledge is usually presented using laws, concepts, patterns, rules, etc. However, the original data for knowledge acquisition is usually semistructured or structured and may also be distributed in different data network structures, which greatly increases the difficulty of knowledge discovery. With the development of web technology, knowledge in the information field is also accumulating, and extracting valuable information from a large amount of data has become an important research focus [24]. Data mining is produced in response to this trend, and it is a management and analysis technology of data, which is an important means of knowledge discovery. According to different application scenarios, it usually includes different aspects of knowledge discovery, such as data classification, association analysis, prediction of temporal patterns, clustering, and deviation analysis.

The second step is to establish a data mining model, which is the core step of the whole data mining based on the existing data mining algorithms, combined with the realistic task requirements, to establish a data mining kernel model. In the process, first, determine the type of task and select the appropriate mining algorithm, then carry out the optimization of algorithms or algorithm combination, and finally carry out experimental verification. The goal of the whole process is to find hidden and valuable information from a large amount of data to provide us with more benefits, as shown in Figure 1.

Typically, decision trees are constructed to generate decision trees based on the probability of occurrence in certain situations, and it is a decision tree method for assessing project risk; moreover, it is a graphical method using probability analysis. The decision tree is constructed by first training the sample set and by classifying the sample set to produce the final set of decisions [25]. Overall, the final decision tree is a decision set consisting of a tree structure, whose leaf nodes represent attribute class names, the leaf nodes connected to the decision root node represent a classification, and the path between the decision root node and the leaf nodes represents the classification rules of the attributes.

The best way to understand the current state of classroom teaching and to solve problems in the classroom is to research classroom teaching. Whether it is a smart classroom or a traditional classroom, there are still some problems and needs in the classroom teaching of junior high school English. Classroom observation provides a holistic view of classroom teaching and learning, as well as an understanding of the interactions between the various components of the classroom. Video analysis is used to analyze the video recordings of classroom teaching and learning and to reflect the overall characteristics of teaching behaviors in the classroom in an objective way. The work of teachers is characterized by professionalism and complexity, and they are the transmitters of knowledge.

### 2.2. Data

In this study, a search on CNKI with TPACK as the keyword yielded a total of 1079 articles, and the distribution of the main topics of TPACK domestic research is shown in Figure 2. The topic distribution chart shows that the most domestic ontology studies on TPACK are found, with 773 articles, which is more than half of the weight. The next is the research on teacher-training students, which includes the survey on the current situation of TPACK for teacher-training students, the factors influencing TPACK for teacher-training students, and the research on the improvement strategies and information ability of teacher-training students in the framework of TPACK. 50 articles were published, accounting for 3.60% of the total. Next is the research on disciplinary pedagogical knowledge of integrated technology, including the research on TPACK of teachers of different disciplines and TPACK of teacher-training students [26]. It creates a novel and relaxed classroom atmosphere, attracts students' interest in learning, and improves students' learning motivation. In the information teaching ability, the main research is on the investigation of the current situation of preservice and in-service teachers' information ability in the context of information technology and the study of ability enhancement strategies.

The basic research mainly includes the introduction of TPACK research progress at home and abroad, the connotation and characteristics of TPACK, and the influencing factors. Applied research is the most active part of the research, including TPACK-based framework subject teaching, teacher training, and in-service teacher training. The TPACK-based framework promotes the integration of information technology and subject curricula and facilitates curriculum reform. The status quo survey is mainly to study the current TPACK level of teachers, the difference of TPACK level of teachers in different areas and different regions, and the difference of TPACK level of teachers in different stages of teaching [27]. The rule of coding classroom behavior mentioned in the Flanders interactive analysis system is to code samples in units of 3 seconds. However, in the real teaching process, the teaching behavior cannot last for 3 seconds, which may cause the continuous unit to be redundant and unnecessarily difficult. Developmental research includes research on the development of TPACK among teacher trainees and in-service teachers, using both qualitative and empirical research methods. Evaluation research is also an important research issue that can be used to promote the continuous improvement and development of the TPACK framework as well as provide developmental suggestions and strategies for the improvement of teachers' TPACK knowledge through feedback, as shown in Figure 2.

Since video analysis is an actual recording of classroom teaching, it can be played in an infinite loop, and it can also be viewed from different angles of the actual video recording, which is free from the limitation of time. When the researcher conducts video analysis, he can adjust the playing time and speed of the video at any time according to his progress, and he can see the small parts more clearly and distinctly. In addition, compared with live coding, the results obtained from video analysis are more realistic, and teachers are affected by the external environment in classroom teaching, so reducing external interference is conducive to more realistic feedback of results.

Next, the selected smart classroom and traditional classroom videos were coded concerning the teacher teaching behavior coding table and TPACK coding table. Before encoding the videos, the classroom videos were processed and the irrelevant instructional content was removed with the help of video editing tools. The video is encoded using video software, and the formal encoding is performed by precoding to test the reliability and validity and to modify any problems that arise [28]. Second, the behavior that occurs more frequently is asking questions. According to the classroom teaching video, it is mainly the teacher who asks questions about the content of the classroom teaching. After that, the video coding is visualized and the data of smart classrooms and traditional classrooms are classified and organized to calculate the timeshare and average frequency of behaviors.

Different researchers conducted empirical studies based on this coding, which proved the validity and scientific of this coding sheet and provided a research tool for conducting classroom teaching video analysis in the information technology environment. In this study, teachers' teaching behaviors were coded and analyzed from five aspects with the help of this coding sheet as a research tool. The continuous state unit recording method was used in conducting the coding to make the teachers' teaching behaviors complete and facilitate the recording and analysis of the coding, as shown in Table 2.

The coding rules and coding sheets were revised and improved in response to the problems that arose during the trial coding process, and finally, the TPACK coding sheets and coding rules were determined through the guidance of educational technology experts. Although the coding rules are an important basis for coding, in the actual coding process, not only the teacher's teaching events, i.e., discourse, should be considered, but also the role of students and the use and role of media technology in this teaching process.

The forms record the start and end time of each coding unit, the category of teachers' teaching behaviors, the media usage, the codes of each TPACK element, and the notes [29]. Notes can record the corresponding instructional content and instructional events. The duration of each behavior can be seen through the teacher's teaching behavior and TPACK record form.

Before recording and analyzing the classroom video coding in two different classroom environments, we first watched the sample videos and used video editing tools to delete the parts that were not related to the teaching content, such as the presentation of the topic before the teacher formally taught, the introduction of the teacher's information, and the redundant recorded parts that were not related to the classroom teaching at the end of the course. This was followed by TPACK at 27%, PCK at 18%, TPK at 17%, and CK and TK with a smaller percentage of duration. The video was positioned to the part related to the teaching content as the beginning of the instructional video.

Then, the timeshare of specific behaviors was calculated: the frequency and total duration of each behavior in each sample were counted separately, and the ratio of the total duration of each behavior to the classroom length in each sample was calculated, i.e., the timeshare of behaviors, and its average value was obtained; for TPACK data, the timeshare and average frequency of each element of TPACK were calculated as the same process of teacher teaching behavior data analysis [30].

## 3. Result

Teachers should have different strategies to respond to the above characteristics. For the phenomenon of students' inability to understand concepts, teachers can introduce concepts by creating situations, demonstrating experiments, and asking heuristic questions to promote students' thinking and understanding. For students who do not know how to use certain methods of inquiry, teachers can increase the number of hands-on opportunities for students, emphasize the use of the scientific method in demonstration experiments, and continuously improve students' ability to use the methods of inquiry through each inquiry activity. For the physical phenomenon is not close enough to the school, teachers should not only make the physics knowledge and life as far as possible.

In response to students' inability to systematically integrate knowledge, teachers should pay attention to the assimilation of old and new knowledge in teaching and be good at helping to guide students to assimilate new knowledge with old knowledge to promote knowledge transfer, as well as to improve students' ability to systematically integrate knowledge. Therefore, for the object of this practice, the integration of receptive learning and inquiry learning should be carried out with deep consideration of the psychological characteristics of students, and different teaching methods should be flexibly selected to adjust the ratio of receptive and inquiry according to the different problems that arise when students learn physics. If students are more suitable for the receptive learning style, then let acceptance take up a larger proportion and vice versa and increase the component of inquiry.

### 3.1. Analysis

Through the statistical analysis, the frequency and duration of each element of senior teacher A's TPACK were made into a bar chart and a fan chart, as shown in Figure 3. In terms of the frequency of each element, the most frequent element in teacher A's TPACK structure was TPK, followed by TCK, PCK, and TPACK, while CK and PK appeared less frequently in the teaching process. In terms of the duration of each element, the longest duration is TCK, which accounts for 31% of the total duration of the course, followed by TPACK at 27%, PCK at 18%, TPK at 17%, and CK and TK at a smaller percentage of the duration. The statistical results show that teacher A is good at explaining the content through technology and pays attention to the effective integration of subject knowledge. The results show that teacher A is better at explaining the content through technology and focuses on the effective integration of subject knowledge, pedagogy, and technology to improve students' learning efficiency and ensure the successful completion of teaching tasks. For the fact that physical phenomena are not close enough to junior high schools, teachers should not only combine physical knowledge with real life as much as possible but also cultivate students' abstract thinking ability.

In terms of the frequency of each element, the most frequent element in the TPACK structure of senior teacher B was PCK, followed by PK, TCK, and TPACK, while CK and TK appeared less frequently in the teaching process. In terms of the duration of each element, the longest duration is the TCK element, which accounts for 44% of the total duration of the course, followed by PCK at 23%, TPACK at 16%, PK at 10%, and CK and TK at a smaller percentage of the duration. The statistical results show that teacher B focuses on the integration of subject knowledge and pedagogical knowledge, is good at promoting students' learning through various teaching methods, and focuses on the integration of technology to help students learn better and improve teaching efficiency. The results show that teacher B focuses on the integration of subject matter knowledge and pedagogical knowledge and is better at facilitating students' learning through multiple teaching methods, as well as integrating technology to help students learn more effectively.

In the dual context of the information technology era and the postepidemic era, blended teaching has also been well developed at the school. However, as the application of the blended teaching model continues to grow, the implementation effect of blended teaching has also attracted much attention, thus revealing many problems. In this study, the effectiveness of English teachers' teaching behaviors in the context of blended learning and teaching was investigated.

Teachers can assign independent learning tasks to students according to their teaching objectives and progress, but few of them give clear output goals. However, the difference is that school English teachers assign fewer online learning tasks and rely mostly on face-to-face classroom instruction. In terms of analyzing online learning data, most teachers neglected to analyze and summarize online learning data.

### 3.2. Relevance

By longitudinally observing the frequency of the PCK elements in the classroom teaching behavior categories of the four teachers, it was found that the PCK elements were mainly reflected in the classroom teaching behaviors of asking questions, giving instructions or directions, and interacting. Remarks can record the corresponding teaching content and teaching events. The duration of each behavior can be clearly seen through the teacher teaching behavior and TPACK record sheet. As shown in Figure 4, the frequency of interactive behaviors was the highest. According to the classroom video, the interaction is done jointly by teachers and students, mainly in the form of one question and one answer, which makes the classroom learning atmosphere more relaxed and can guide students' thinking and help them consolidate their knowledge. Second, the more frequent behavior is questioning. According to the classroom video, the teacher mainly asks questions about the classroom content to improve students' concentration on the learning content and to test their knowledge proficiency. According to the classroom video, the teacher gives instructions or directions in theory courses mainly when students are browsing resources or having group discussions and in practice courses mainly when students are creating work. According to constructivist theory, the teacher is the guide of students' learning, so it is very important to give appropriate guidance or instructions to students during the teaching process, not only to prompt students' thinking but also to encourage or correct students' ideas in time.

The horizontal coordinates are the eight teacher control behavior codes and the seven student control behavior codes corresponding to the classroom teaching behavior classification, and the vertical coordinates are the duration of each element of TPACK in the teacher's classroom teaching behavior. The duration of each element in each teaching behavior and the different colors in each teaching behavior represent the elements of TPACK associated with that teaching behavior.

The stacked bar chart shows that school IT teachers' classroom teaching behavior classification has a high proportion of TPACK and TCK elements, which are mainly reflected in classroom teaching behaviors such as giving instructions or directions, interacting, and explaining. This indicates that school IT teachers are good at using technology for classroom teaching, and they are good at integrating technology with other elements in TPACK in the form of composite elements. The original data for knowledge acquisition is usually semistructured or structured and may also be distributed in different data network structures, which greatly increases the difficulty of knowledge discovery. Teachers rarely used only technology in the classroom teaching process, and subject knowledge did not rely exclusively on technology for transmission. In addition to the explanation of subject knowledge, students are also instructed or interacted with by teachers and students through technology. When learning in such a relaxed and harmonious learning atmosphere, students are more interested in learning and their learning efficiency is improved.

As grade levels change, learners grow older, and learners' knowledge related to IT subjects changes, learners' learning styles change, and their need for emotional feedback from teachers changes, so senior year, teachers pay more attention to supporting students emotionally and enhancing their confidence in learning high school IT at the beginning. Teachers will be affected by the external environment in classroom teaching, so reducing external interference is conducive to more realistic feedback. The classroom behaviors of sophomore IT teachers included a more frequent and longer duration of explanation and interaction than those of first-year IT teachers. Sophomore students have a certain foundation for school IT courses and have mastered the relevant learning methods, so teachers can make students learn more easily through interaction. At the same time, the IT courses in the sophomore year are more difficult than those in the first year, and the frequency and duration of teachers' classroom teaching behaviors have increased.

Theoretical courses are mainly learning the basic theoretical knowledge of IT subjects, which does not mean that teachers in the courses do not use technology or do not allow students to deepen their understanding of basic theoretical knowledge through technology; operational courses are mainly learning operational skills of IT subjects, which does not mean that teachers in the courses only teach technology without teaching students the theoretical basis of technology operation. In the teacher control dimension, IT teachers explained more frequently in the process of teaching operational courses than in teaching theoretical courses. This indicates that teachers teach operational courses with a great deal of supplementary explanation to give students a better and more comprehensive grasp of the basics of operational skills. The frequency and duration of instructions given by the IT teachers in the process of teaching manipulative courses were greater than that of teaching theoretical courses. In the process of teaching manipulative courses, teachers needed to guide students or aid in the process of students' independent manipulation, as shown in Table 3.

Proficiency in the use of multiple pedagogical approaches is essential to be a school IT teacher. The statistical results showed that the dimensions related to pedagogical knowledge in TPACK were present in almost the entire classroom, both in terms of frequency and duration. It is also clear from the classroom videos that all four teachers have mastered a variety of teaching methods and can select the appropriate teaching method according to the content. The use of multiple teaching methods in the actual classroom teaching process can improve students' learning efficiency, deepen students' memory of knowledge, and cultivate students' independent thinking and teamwork skills.

The subject pedagogy knowledge of integrated technology is a new requirement for school IT teachers in the information technology era. The statistical results show that a high percentage of school IT teachers use the subject pedagogy knowledge of integrated technology in the classroom teaching process, which indicates that school IT teachers can keep up with the development of the times and update their knowledge structure. According to the classroom teaching videos, teachers infiltrate technology in teaching behaviors such as explaining, asking questions, giving guidance or instructions, interacting, and praising or encouraging, creating a novel and relaxed classroom atmosphere that attracts students' interest in learning and increases their motivation to learn.

As observed in the classroom, the act of asking questions is one of the main aspects of teacher-student interaction in traditional classrooms, and it is also a way to help teachers conduct follow-up checks to test students' understanding and application of knowledge. There are differences in teachers' TPACK levels in different fields and regions and teachers' TPACK levels in different stages of teaching. However, in the smart classroom environment, the teacher's questions are not only limited to the act of asking questions, but the teacher can deliver the questions to the students in different forms, for example, the teacher can use the teacher-side and student-side intercommunication function to send the questions directly to the students' tablets, and the students can operate on the tablets and then send out the answers.

The performance is a sequence of question-student-initiated speech-praise and question behavior, which can make students have a deeper understanding and mastery of a certain knowledge point; when students make a speech or presentation, due to students' expression level or personal factors such as nervousness, which leads to a short silent behavior during the speech or presentation, the arrow between students making a presentation and speech and silence or chaos in the figure is two-way, and the sequence of behavior. This indicates that teachers pay more attention to the main position of students in classroom teaching and arrange students to make learning presentations, but this approach also makes it easier to make the classroom appear silent and chaotic and other uncontrolled behaviors due to students' inadequate preparation. The arrow between students' collaboration and giving guidance and instructions is a two-way arrow, which indicates that teachers can give timely guidance and help to students for the problems or situations they encounter in the process of collaboration in the classroom. The arrow between students using educational resources and giving instructions is a two-way arrow, indicating that students encounter different problems in the process of using media resources.

## 4. Discussion

Teacher questioning-interactive facilitation or emphasis-explanation-questioning-student-initiated speaking acceptance or use of student claims differs from the previous behavioral sequence in that the teacher asks questions followed by student-initiated speaking and accepts and uses student claims. This process focuses on the teacher asking the question again toward hearing the student's response and the teacher accepting the student's response or exploring more deeply through the student's response after the student has answered correctly. We can see that teachers in smart classrooms pay more attention to the dominant position of students, and teachers pay more attention to cultivating students' autonomous learning ability and group nature. The teacher gives full play to the role of a mentor in the organization of teaching activities, giving timely guidance to students in the learning process and helping them to complete learning activities and solve learning difficulties.

## 5. Conclusion

Student behaviors and teacher-student interaction behaviors were lower in the percentage of time and frequency of occurrence, and silent behaviors were present in both classrooms. The difference is that from the traditional classroom to the smart classroom, the teacher's teaching behaviors have changed somewhat. In the teacher behaviors, the time spent on explaining and questioning behaviors decreased, and the time spent on giving instructions and directions and on practical activities with the help of media increased, and the total time spent on teaching behaviors decreased. The overall time and frequency of student responses decreased in student behaviors, aphysics, and it is also effective in changing some students' attitudes toward physics and increasing the time and frequency of student demonstrations and speech act, and student creative work acts increased significantly. Two classification prediction models, the cluster-then-classify model and the cluster-classification integrated model, were used. These two models used the algorithm to fine-grained the data set from the perspective of subject users and mental health factors, respectively, and then used the decision tree algorithm to classify and predict the mental health factor information from the subject user base information. In terms of media behavior, the types of instructional media and the functions of instructional media were diversified, and the teachers' media manipulation behavior also became diversified. The integrated teaching method is effective in improving students' performance in their self-confidence in learning physics.

## Figures and Tables

**Figure 1:** Psychological data analysis framework.

**Figure 2:** Theme distribution map.

**Figure 3:** The proportion of time spent on each element of teacher A's TPACK.

**Figure 4:** Relevance results.

**Table 1:** Rules for coding classroom teaching behaviors.

Dimension	Serial number	Content	Behavior
Classroom teaching behavior dimension	1	Acceptance and positive feelings	Teachers
	2	Praise or encouragement	
	3	Accept or use student claims	
	4	Ask questions	
	5	Students give speeches (especially in front of teachers)	Students
	6	Student collaboration	
	7	Students browse resources or think about problems independently	
	8	Students create work (e.g., composition and programming)	

**Table 2:** Faculty teaching behavior coding.

Dimension	Serial number	Content
Classroom teaching behavior dimension	B 1	Students give speeches (especially in front of teachers)
	B 2	Student collaboration
	B 3	Students browse resources or think about problems independently
	B 4	Students create work (e.g., composition and programming)
	B 5	Acceptance and positive feelings
	B 6	Praise or encouragement
	B 7	Accept or use student claims
	B 8	Ask questions

**Table 3:** Adjusted residuals.

Coding	B 1	B 2	B 3	B 4	B 5	B 6	B 7	B 8
B 1	0.477	0.579	0.764	0.992	0.954	0.658	0.534	0.591
B 2	0.899	0.449	0.857	0.945	0.922	0.462	0.884	0.61
B 3	0.958	0.662	0.786	0.514	0.958	0.43	0.422	0.895
B 4	0.615	0.656	0.88	0.987	0.493	0.725	0.989	0.579
B 5	0.598	0.741	0.506	0.997	0.872	0.69	0.78	0.403
B 6	0.811	0.485	0.871	0.7	0.461	0.421	0.877	0.567
B 7	0.986	0.812	0.901	0.541	0.631	0.739	0.781	0.666
B 8	0.581	0.8	0.445	0.534	0.909	0.589	0.46	0.906

## Data Availability

The data used to support the findings of this study are available from the corresponding author upon request.
